# Load-Balancing Strategy: Employing a Capsule Algorithm for Cutting Down Energy Consumption in Cloud Data Centers for Next Generation Wireless Systems

**DOI:** 10.1155/2023/6090282

**Published:** 2023-02-20

**Authors:** Jyoti Singh, Jingchao Chen, Santar Pal Singh, Mukund Pratap Singh, Montaser M. Hassan, Mohamed M. Hassan, Halifa Awal

**Affiliations:** ^1^College of Information Science & Technology, Donghua University, Shanghai, China; ^2^Department of Computer Science & Engineering, Rashtrakavi Ramdhari Singh Dinkar College of Engineering, Begusarai, India; ^3^School of Computer Science Engineering & Technology, Bennett University, Greater Noida, India; ^4^Department of Biology, College of Science, Taif University, P.O. Box 11099, Taif 21944, Saudi Arabia; ^5^Tamale Technical University, Tamale, Ghana

## Abstract

Per-user pricing is possible with cloud computing, a relatively new technology. It provides remote testing and commissioning services through the web, and it utilizes virtualization to make available computing resources. In order to host and store firm data, cloud computing relies on data centers. Data centers are made up of networked computers, cables, power supplies, and other components. Cloud data centers have always had to prioritise high performance over energy efficiency. The biggest obstacle is finding a happy medium between system performance and energy consumption, namely, lowering energy use without compromising system performance or service quality. These results were obtained using the PlanetLab dataset. In order to implement the strategy we recommend, it is crucial to get a complete picture of how energy is being consumed in the cloud. Using proper optimization criteria and guided by energy consumption models, this article offers the Capsule Significance Level of Energy Consumption (CSLEC) pattern, which demonstrates how to conserve more energy in cloud data centers. Capsule optimization's prediction phase F1-score of 96.7 percent and 97 percent data accuracy allow for more precise projections of future value.

## 1. Introduction

Cloud computing is an extension of grid, parallel, and distributed computing techniques [1]. To achieve cloud computing, it conveys an assortment of equipment administrations, framework administrations, stage administrations, program administrations, and capacity administrations over the Web. Clients of cloud computing can utilize it on-demand, pay for it on-demand, and scale it up and down easily. Data centers have grown in size as cloud services have grown in popularity, necessitating a considerable amount of energy consumption. The authors pointed out in [2] that data centers consume 1.5% of the yearly control created within the assembled states, agreeing with insights from the US Division of Energy. China's data centers are projected to consume about the same amount of energy as the United States and have surpassed the Gorges' yearly power generation. The estimation of energy consumption has become the most difficult challenge in today's data center, so reducing energy consumption is a pressing issue that needs to be addressed in cloud computing research. One of the most predominant ways of bringing down vitality utilization is virtual machine solidification. The overload/underload location, virtual machine determination, virtual machine arrangement [3–5], and virtual machine relocation [6, 7] are all cases of positive virtual machine combination. Virtual machine movement can take a long time, squander a part of assets, and meddle with the working of other virtual machines on the server, resulting in a decrease in framework execution. Virtual machine relocation too requires the utilization of additional organized capacity [8]. The detailed descriptions of energy consumption architecture and data flow are given below in Figure 1.

Virtualization is an important method in data centers because it allows customers to share resources by using virtual machines (VMs). Each virtual machine is separated and utilized to run customer applications, with storage capacity, primary memory, CPU, I/O capabilities, and network bandwidth requirements [9]. Some of the important characteristics that promote cloud computing performance are physical machine consolidation, fault tolerance, and load balancing. Physical Machine (PM) consolidation occurs through Virtual Machine (VM) migration, which occurs when a virtual machine's requested resources are unavailable on the physical machine, causing the virtual machine to be relocated. The VM is moved to another physical computer to meet the VM requirement [10]. The suggested method forecasts the power of each VM before VM migration, and then VMs are migrated to certain PMs based on this prediction and resource availability. The VM power prediction improves system availability, reduces infrastructure complexity, and lowers cloud providers' operational costs, allowing customers to pay less [11]. To manage operations faster and deliver more reliable services to clients, it is necessary to forecast the VM's power in advance. Power conservation can be achieved by using various machine-learning approaches to forecast power use. This machine-learning-based technique is used in this study to forecast virtual machine power consumption, enrich cloud computing infrastructure, and improve service for IT industries. Furthermore, the power consumption of virtual computers is forecasted before they are assigned to physical machines [12].

The proposed technique is exceptionally good at finding acceptable computer resources in unknown networks since it incorporates a great positive input instrument and a dispersed look strategy. This article has provided a user-experience-based procedure for finding energy-saving virtual machines. The strides roulette likelihood choice component guides and maintains a strategic distance from the calculation entering the basic information to untimely joining, viably decreasing vitality utilization, and accomplishing an adjustment between vitality utilization and client encounter by altering the pheromone and heuristic calculate upgrade strategies and characterizing the parameter administrative calculate. Cloud information centers offer various benefits, including on-demand assets, elasticity, flexibility, portability, and calamity recuperation [13]. One of the most important aspects of the cloud worldview is adaptability, which enables an application to grow its asset requests at any time [14]. Instead of purchasing and controlling computing resources, it has become more common to rent hardware, software, and network resources. With an Internet connection, users can take advantage of the entire processing infrastructure. It can be used in a wide variety of contexts, including commercial management, academic research, hospital administration, manufacturing, marketing, and many more [15].

The following is our contribution:

- Using historical data, we investigate and analyze the energy use of the data center. The results of this article are utilized to create a statistical model that links meteorological variables to energy use.
- To use the statistical model to create a forecast model that can predict the data center's energy usage based on the weather forecast. The model is validated by comparing it to real-world resource usage data obtained using the capsule optimization technique.
- To provide data center operators with an energy consumption forecast technique that allows them to optimize their power distribution and energy consumption by providing estimations of their resource utilization.

The structure of the paper is laid out underneath.  Section 2 has literature from past inquiries about workload estimation and vitality utilization in a cloud information center. The proposed framework for controlling utilization based on ML-based approaches is examined in Section 3.  Section 4 depicts the proposed approach's performance evaluation and serves as a conclusion in Section 5.

## 2. Literature Review

In the context of cloud server energy consumption management, the background of research, such as CPU utilization forecasting and resource usage forecasting and management, is one of the most successful techniques for anticipating the future. The amount of power required to run and cool down the devices in the cloud data center increases day by day, increasing cloud service providers' operational costs. For better performance of a complex function, power consumption prediction is utilized to estimate the nonlinear future value. In [16], the author discussed an adaptive threshold method, local regression, and robust local regression to evaluate overloaded servers in IaaS infrastructure based on CPU use. The threshold is automatically changed based on previous data analysis and manipulation with estimators such as mean absolute deviation and interquartile range. The author [17] focused on applying autoregressive linear prediction to anticipate network demand. In this strategy, the data samples utilized for training to discover the link between attributes were smaller using cross-validation and the black box method. The author in [18] introduced a tree regression (TR)-based model to compute VM power usage. The black box method is used to collect information on the VM and server features. For their prediction model, they used data as linear values. The author discussed the linear regression approach for forecasting cloud service workload [19]. They also used the auto-scaling technique to lower the operational costs of virtual resources by scaling them both vertically and horizontally. Using NASA trace and Saskatchewan trace, we devised a self-adaptive differential evolution algorithm to estimate the workload used by the cloud data center in [18]. The author discussed fitness function, mutation, and crossover in this method, which they found to be superior to other approaches such as particle swarm optimization (PSO), genetic algorithm (GA), and others.

In [20], the author discussed three versatile models for high vitality utilization and infringement of service-level understandings. When selecting virtual machines from overburden to decrease vitality utilization, SLA infringement was taken into consideration. At the same time, the execution of cloud information centers can be ensured. In [21], the author discussed the models for diminishing the vitality utilization of portable cloud information centers amid periods when virtual machines are inadequate or overburdened. For virtual machine determination and energetic blending, the recommended versatile heuristic energy-aware calculation perceives the history of CPU usage, which diminishes add up to vitality utilization and improves benefit quality. Compared to the most existing research, in [22], the author explored two extra key variables while handling the challenges of cloud data center energy usage and SLA violations: (1) Examining the stability of the CPU consumption upper limit. (2) When picking the virtual machine of the overburden based on the CPU utilization expectation, the execution debasement time and SLA infringement are diminished. To decrease vitality utilization with negligible SLA taking a toll, a heuristic method is displayed to identify the least-squares relapse of the overburden and select the virtual machine from the overburden with the lowest utilization estimate. In [23], the author discussed an energy-aware energetic virtual machine choice calculation proposed in [23] for the issue of virtual machine integration to coordinate virtual machines from overburdened or underloaded to upgrade vitality utilization and expand benefit quality. There are a few pieces of literature listed below in Table 1.

In [31], the author discussed the problems of reducing VM power usage and cloud vendor operational costs in a cloud setting. They used an ad-hoc framework for VM consolidation, but this method ignored VM requirements such as disc space, network bandwidth, and the time it took a VM to execute a task. The author has suggested [32] the use of a radial basis function (RBF) neural network to examine the power of VM with normalized parameters that satisfy the correlation coefficient of VM's power. This method used a tiny amount of samples for training and testing data, resulting in a neural network that could not make an accurate prediction. In [33], the author used machine learning methods to estimate VM resource management in the cloud platform based on Azure workload parameters such as first-party IaaS and third-party PaaS services. The authors used the fast Fourier transform to determine the type of VM workload and the cumulative distribution function to produce the graphs for CPU, memory, CPU core utilization per VM, and VM lifetime. After each prediction, accumulate the results in the Dynamically Linked Library (DLL) and determine whether the forecast was worthwhile. In [34], the author used supervised learning algorithms to analyze the workload of VM to reduce its power consumption. They compiled a list of different scheduling strategies for reducing carbon dioxide emissions from a data center. The prediction error was calculated using statistical metrics such as RMSE, R squared, and accuracy, which were calculated using an algorithm. The recurrent neural network was used to forecast and manage resource allocation to a cloud server. They used time-delay neural network (TDNN) and regression approaches to compare the outcomes of the server workload prediction. In [35], an adaptive selector neural network was developed for selecting the strategy for active VM reduction, and the results were compared to those of linear regression. The customer's Service Level Agreement (SLA) with the cloud service provider was also crucial to this strategy; however, SLAs are still not met when customer requirements change. The contribution of this study is also found in the description of a load-balancing algorithm inspired by energy consumption patterns that shows how we may save more energy in cloud data centers by using appropriate optimization rules informed by our energy consumption models in the literature.

## 3. Proposed Methodology

The points of interest of the proposed demonstration counting preprocessing step and demonstration portrayal are given in the following segment. The proposed model and data flow are given in Figure 2. This work has been gathered from input requests from a user and includes data cleaning, data balancing, transformation, aggregation, and data normalisation in the data preprocessing steps of the proposed model.

The estimation of energy consumption uses a machine learning data model, which has been included in a Capsule algorithm that drops out fully connected layers. The cross-entropy has been calculated using the Softmax layer. The evaluation metrics are calculated using the proposed model and compare the accuracy of the model with the state-of-the-art models (ant colony and random forest).  Figure 3 depicts a visual representation of the data center.

The request of a user has to supply in two ways request such as power path to IT and power to secondary support. The data center consisted of an uninterruptible power supply (UPS) and a Paragon Development System (PDS), as well as cabling and cooling light conditions. Furthermore, the data request was transferred to the IT load. There are a few abbreviations given in Table 2.

The data flow of the proposed capsule significance level of energy consumption (CSLEC) is given in the form of a few steps, which are described in Algorithm 1 and Figure 4.

  Step 1: the operational module gets the machine's current working status within the cloud data middle and then performs state control on each host
  Step 2: we exchange the host's running status and virtual machine line state to the client encounter module and obtain the accessible assets based on the CPU use edge you set
  Step 3: within the virtual machine planning module, initialize the pheromone for accessible resources
  Step 4: we put all of the capsules on the accessible at random
  Step 5: the capsule chooses another by calculating the likelihood determination instrument based on the pheromone concentration, the heuristic figure, and the alteration factor
  Step 6: in case the CSLEC algorithm completes the look, upgrade the neighborhood and worldwide pheromones; on the off chance that it does not, return to Step 5
  Step 7: the framework produces the ideal assignment scenario when the number of initialization emphases is met; otherwise, it returns to Step 4
  Step 8: we check to see if there are any virtual machines

The complete steps have been described in Algorithm 1.

The flowchart of the proposed CSLEC model is shown in Figure 4. The data are entered into the host voltage system, where the information is controlled and the profit matrix is calculated. The performance of the host machine is initialized, and if it meets the iterations of the system, then the output is calculated. If it does not meet the requirements, then the capsule model is placed and put in VM after calculating the transition probability with local and global updates.

### 3.1. Fitness Function Design

The suggested technique's main purpose is to provide tighter cloud load balancing. Cloud computing has a certain number of PMs, each of which has a certain number of VMs. The first item in equation (1) stands for control utilization (*P*), the moment term stands for movement taken a toll (MC), and the third term is for memory utilizes (MU). The outright Euclidean separate (ED) of all the energetic PM at the same time determines the framework's power usage. The load-balanced system with the reduced ED is thought to be better. When no assignment is run in the relevant PM, the PM is turned off. The power efficient factor (EF) of each active node is calculated based on equation (2).

(1) $$\begin{array}{c} Fitness\_function=\mathrm{Min}\left(\beta_{1}\left(q\right)+\beta_{2}\left(MC\right)+\beta_{3}\left(MU\right)\right)\text{.} \end{array}$$

The first component in equation (1) stands for control utilization (*q*), the moment term stands for movement taking a toll (MC), and the third term stands for memory utilization (MU). The outright Euclidean separate (ED) of all the energetic PM at the same time decides the framework's control utilization. The load-balanced framework with the diminished ED is thought to be way better. When no task is run within the significant PM, the PM is turned off. Condition is utilized to decide the control proficiency figure (EF) of each dynamic hub equation (3).

(2) $$\begin{array}{c} E_{F}=\sqrt{\overset{d}{\underset{k=1}{\sum }}}{\left(V-VBest_{i}\right)}^{2}\text{,} \end{array}$$

where *i*⟶ Memory resources. *Vi*⟶ Given resource utilization. *V*Best_*i*_ ⟶Best utilization of resource *i* for power efficiency in each physical node.

Power efficiency at time *t* is calculated as follows in equation (4):

(3) $$\begin{array}{c} PT=\sum EF\text{.} \end{array}$$

System total power efficiency is represented as

(4) $$\begin{array}{c} P=\overset{T}{\underset{t=0}{\sum }}E^{t}\text{.} \end{array}$$

Another consideration for the objective function is the cost of migration. When the number of motions increases, the MC of the VM expands. The best load-balancing system should have the least amount of movement. The MC of the entire cloud arrangement is calculated using the conditions provided in

(5) $$\begin{array}{c} MC=\frac{1}{V}\overset{v}{\underset{i=1}{\sum }}\left(\frac{No\_of\_migration\_in\_VM_{s}}{Total\_no\_of\_VM_{s}}\right)\text{.} \end{array}$$

Another aspect of the load-balancing target function is memory use. Memory is nothing more than a jumble. The heap structure is honestly based on the VM's benefits for setting up the assignments from various customers. CPUs and memory storage are among the resources used by the VM. The storage utilization of the entire cloud setup is calculated using conditional logic equation:

(6) $$\begin{array}{c} MU=\frac{1}{PM\times VM}\left[\overset{PM}{\underset{i=1}{\sum }}\overset{VM}{\underset{j=1}{\sum }}\frac{1}{2}\left(\frac{CPU\_Utilization_{ij}}{PU_{ij}}+\frac{Memory\_Utilization_{ij}}{Memory_{ij}}\right)\right]\text{.} \end{array}$$

In condition (1), the objective work of our investigation is indicated. In this paper, the overobjective work is getting to be minimized by utilizing the ACSO calculation.

#### 3.1.1. Data Balancing

The class imbalance problem happens when the quantity of samples in distinct classes of a dataset is unequally distributed. Minority classes receive fewer samples than other target groups, whereas majority classes receive more samples [36]. Minority classes must be properly supplemented since they are crucial for extracting information from unbalanced datasets. A method for boosting the sample size of minority groups is the Synthetic Minority Oversampling Technique (SMOTE). Using this technique, new artificial samples are produced next to existing samples and then arranged in a line. After that, samples from nearby minority groups are matched with them. Notably, the sample features in adjacent classes are unaffected, permitting SMOTE to create tests that drop interior with the most dispersion. The recently made counterfeit information, which is calculated and utilized, is

(7) $$\begin{array}{c} D_{new}=D_{i}\left(D_{l}^{*}-D_{i}\right)\times \delta \text{.} \end{array}$$

It is a number between 0 and 1, where *D*_*i*_ represents the number related to minority samples and is the closest neighbour. The capacity to generate new samples close to minority class data is one of the SMOTE technique's most noticeable advantages over other resampling techniques. This strategy is less complex and simpler than other data-balancing methods like cost-sensitive ones.

### 3.2. Feature Transformation

In our suggested model, label encoding is employed to convert nominal properties into numeric ones that may be interpreted by neural networks. Label embedding takes into account a number between zero and *n*−1 for each sample with nominal properties [18]. The reason for using this strategy is that it does not alter the data's dimensionality.

#### 3.2.1. Data Aggregation

It envelops methods that result in the creation of modern highlights by combining two or more existing features. In comparison to the first highlights, the modern highlights must be able to specify the dataset's data more successfully and totally. The proposed work employments information accumulation to decrease dimensional whereas moreover expanding the value of highlights and information soundness [20].

#### 3.2.2. Normalization

The suggested model normalises the input data using the Max-Min normalisation method. This method applies a linear change to the original data while preserving the correlation between them [13]. The normalisation approach is employed because the relationship between independent variables and the correlation between data are important in the prediction stated in

(8) $$\begin{array}{c} X\left(n\right)=\frac{x-\mathrm{Min}\left(A\right)}{\mathrm{Max}\left(A\right)-\mathrm{Min}\left(A\right)}\text{,} \end{array}$$

where Min(*A*) and Max(*A*) denote the feature's minimal and maximum values, respectively, and *x* denotes the feature's current value.

### 3.3. Proposed Model

A capsule may be a collection of neurons whose movement vector speaks to the instantiation parameters of a specific sort of substance, such as a protest or a question parcel [14]. To put it another way, capsules encapsulate in vector form all relevant information about the status of the feature they are detecting [18]. Since the capsule is a vector, the length of it is a probability of detection of a feature, which means that even if the detected object has rotated, the length of the vector will be the same (the probability still stays the same), but the vector direction will change in the direction of the change. For example, let's assume that the current capsule has detected a face within an input image with a probability of 0.9. When the face starts to change location across the image, the capsule's vector will change direction, which means that it still detects; however, the length will be the same. This is exactly the form of invariance, which is not the max-pool offer in CNN.

#### 3.3.1. Fully Connected (FC) Layer

Fully linked layers in neural networks are ones where all of the inputs from one layer are connected to each enactment unit of the following layer. Most common machine learning models' final few layers are complete related layers that combine the data retrieved by earlier levels to produce the final result [15]. A “Fully Connected (FC)” layer is planned to proficiently handle vector information. The model's depth should be properly calculated. We used one layer of fully linked layers in this example, but a service provider can alter it to establish a balance between the target model's complexity and the complexity of the target model (better detection accuracy).

#### 3.3.2. Dropout Layer

To avoid overfitting, the dropout layer is used. Dropout is a neural network regularization strategy that reduces recurrent learning between neurons. As a result, certain neurons are disregarded at random during the training process [18].

#### 3.3.3. Classification Layer (Softmax)

In the last layer, Softmax is utilized to categorise the data. The last classification layer of a neural network uses a nonlinear activation function called Softmax [5]. Softmax is calculated using equation (9), and the output values are normalized so that the sum of the values is one.

(9) $$\begin{array}{c} P\left(Y=K,X=x_{i}\right)=\frac{e^{sk}}{\sum_{j=1}^{m}e^{sj}}\text{,} \end{array}$$

where *k* is the conventional exponential function applied to each element of the input vector and is the *k*-dimensional input vector. The fraction's denominator guarantees that all output values are between 0 and 1. The relevant class's score must be maximized in the next section.

## 4. Result and Discussion

This work has provided a comprehensive analysis of energy-saving calculations based on the arrival, processing, and response time of the virtual server. There are two different factors: processor utilization and energy consumption. The experimental evaluation is carried out using the Clouds toolkit. It is a common framework for simulating cloud computing systems on local devices [37]. Cloud components such as data centers, virtual machines, and resource provisioning limits can be simulated using the CloudSim toolkit. Also, for the experiment, choose a sample size of 100 tasks, which were initially distributed over five virtual machines [38].

### 4.1. Evaluation Metrics

The proposed model is evaluated using the accuracy, precision, and recall metrics as given in equations (10)–(12), respectively, where “TP” and “TN” refer to correctly categorized true positive and true negative samples [39]. Positive and negative instances that have been erroneously categorized are also referred to as FP and FN:

(10) $$\begin{array}{c} Accuracy=\frac{TP+TN}{TP+FP+TN+FN}\text{,} \end{array}$$

(11) $$\begin{array}{c} Precision=\frac{TP}{TP+FP}\text{,} \end{array}$$

(12) $$\begin{array}{c} Recall=\frac{TP}{TP+FN}\text{.} \end{array}$$

Table 3 compares the proposed model's accuracy to that of other current models.

The accuracy in Table 3 shows the comparison of different models; the proposed capsule model shows better accuracy in comparison with other pretrained models. This work compares the four different models, such as LR, PSO, Capsule, and CNN, that achieved 70%, 76%, 85%, and 95% data accuracy, respectively [40]. The proposed CSLEC data model has achieved 97% data accuracy, which is better than another model's accuracy. Also, depending on the number of parameters in the trainable stage, the time taken for the training of the proposed model shows a better time in comparison with the pretrained CNN model shown in Table 4.

The accuracy Table 3 shows the comparison of different models; the proposed capsule model shows better accuracy in comparison with other pretrained models. Also, depending on the number of parameters in the trainable stage, the time taken for the training of the proposed model shows better time in comparison with the pretrained CNN model shown in Table 4. The proposed model has been using 25346 trainable parameters, and it has consumed 1577.87 ms of time. This work has compared the four different algorithms: LR, PSO, Capsule network [41], and CNN. The LR algorithm has used 16896 trainable parameters and consumed 588.31 training time. In comparison with the LR model, the PSO model has been used with 17154 parameters and a training time consumption of 946.52 ms. The other training networks, Capsule and CNN, used 20960 and 33410 trainable parameters, respectively, consuming 967.14 and 1702.43 seconds. Out of this basic model, our proposed model has been trained with a large number of data and a 1577.87 consumption rate.  Table 5 shows the difference in energy consumption with the use of different servers in Watts (W). As the level of workload increases, the percentage value of the Hitachi TS10 increases and reaches a maximum of 86.2 watts.

The electric energy consumption has been considered by Fujitsu M1, Fujitsu M3, Hitachi TS10, and Hitachi SS10 server capacities, which has been considered in the range of 0% to 100% workload, and maximum server capacity has been estimated by Hitachi TS10 server as 41 42.9%, 44.3%, 46.6%, 49.9%, 53.9%, 58.9%, 66.2%, 74.9%, 81.9%, and 86.2%. The maximum server capacity and accuracy in Table 5 show the comparison of different server capacities; the proposed capsule model shows better accuracy in comparison with other pretrained models [42]. Also, depending upon the number of parameters in the trainable stage, the time taken for the training of the proposed model shows a better time in comparison with the pretrained CNN model shown in Table 4.  Table 5 shows the difference in energy consumption with the use of different servers in watts (W). As the level of workload increases, the percentage value of the Hitachi TS10 increases and reaches a maximum of 86.2 watts.

The server capacity of this work is shown in Figure 5. The Hitachi TS10 has shown maximum electric consumption. This work has been estimating the electric energy consumption using different four types of servers, such as the “Fujitsu M1,” “Fujitsu M3,” “Hitachi TS10,” and “Hitachi SS10.” Hitachi TS10 [30] has achieved the best energy consumption accuracy of 86.2%. This work has also observed that the Fujitsu M1, Fujitsu M3, and Hitachi TS10 do not provide better energy consumption in terms of watts. The result of the capsule algorithm in the form of different tasks is shown in Table 6.

This work used the task, arrival time, response time, processing time, and energy consumption estimated in the unit of ms. The task has been divided into five different terms, such as T0, T1, T2, T3, and T4. The user request was sent, and the server scheduled it based on the arrival time. The maximum arrival time for task T4 is 22 ms, which is better than other tasks in comparison with processing time. But task T3 takes less processing time in comparison with others and also utilizes the minimum processor with an energy consumption of 54.7. The energy consumed by the considered servers is shown in the form of a graph in Figure 6.

The experiment was double-checked using a larger number of tasks and virtual machines in this paper. The recorded results are also compared in order to assess the research project [43]. The PSO load balancer algorithm is used to parse the simulations, and the results are then logged. The Firefly load balancer is then used to run the same simulations. The findings are analyzed using fixed characteristics such as CPU utilization, reaction time, and throughput [44]. The usage times of both approaches are now calculated using the above-mentioned energy formula. For both the PSO and Capsule algorithms, this yields the energy consumption parameter. The information gathered is analyzed and compared with the algorithms of PSO and Capsule [45]. The information gathered is analyzed and compared [46].

Figure 7 compares the LR, CNN, and PSO models with the proposed model in terms of memory utilization. The proposed model has efficiently provided the accuracy of memory utilization of 170000 nm. The comparative study of the energy consumption is shown in Figure 8.

This project explored a few versions before settling on a few to graphically depict the status. The processing usage of the Capsule load balancer is higher than that of the PSO load balancer [47]. The final parameter for comparing the two algorithms is energy consumption, which is calculated using this utilization [48]. A Firefly load balancer's average response time is faster than a PSO load balancer's. As previously stated, the response time has a wide-ranging impact on energy use. As a result of the faster response time, less energy is consumed [49]. The amount of energy consumed is calculated by employing an equation that utilizes a settled value for the greatest control that can be devoured when the machine is completely stacked and a foreordained value for the least control that will be devoured when the machine is nearly still [50].

## 5. Conclusion

In a cloud data center, energy consumption is a major concern. With the rise in requests and a broad selection of cloud computing, it is presently fundamental to preserve successful and efficient data center methodologies to meet the approaching demands with the slightest amount of assets. In this work, we compared the training parameters and training time of different models, such as CNN, PSO, and Capsule, with the proposed model of CSLEC. The CSLEC model has been used with 25346 training parameters and 1.57 training minutes (ms). The proposed model has achieved an accuracy of 97%. The proposed CSLEC algorithm's mathematical explanation has been thoroughly explained. The experimental outcomes are represented using a variety of measures. In comparison to the existing method, the proposed strategy has the briefest make span and employs the least amount of vitality. In the future, we will actualize our strategy in real time and place a greater emphasis on it. In addition, this work calculated the energy consumed to assess the performance of the Capsule Significance Level of Energy Consumption (CSLEC). Comparative evaluations uncover that the proposed strategy is more successful at optimizing the vitality utilization parameter than the Molecule Swarm optimization calculation. When compared to PSO, the energy consumption of CSLEC is 10–14% lower.

## Figures and Tables

**Figure 1:** Energy consumption architecture.

**Figure 2:** The proposed model.

**Figure 3:** Pictorial representation of data center.

**Figure 4:** Flowchart of energy saving with the CSLEC algorithm.

**Figure 5:** Electric energy consumed by the considered servers.

**Figure 6:** Energy consumed by the considered servers.

**Figure 7:** Memory utilization in the model.

**Figure 8:** Comparative study of energy consumption.

**Algorithm 1:** Capsule significance level of energy consumption (CSLEC).

**Table 1:** Study of energy efficiency methods and algorithms.

Energy efficiency algorithm	Approaches	Weakness	Tools used
Novel resource allocation algorithm for energy efficiency [24]	Autoregressive linear prediction	Energy consumption is not efficient	Power edge
Energy-based scheduling and accounting of VM [25]	Supervised learning methods	High in energy consumption	Simulator (self-designed)
Energy-efficient VM allocation technique using interior search algorithm [26]	Self-adaptive differential evolution algorithm	Maximum the power consumed by data centers	Open-source cloud middleware *Eucalyptus*
Exact allocation and migration algorithm [27]	Adaptive selector neural network	Power consumed by data centers has not reduced and low reduction in the rate of task rejection	Cloud hypervisor xen
Energy-saving VM migration [28]	Linear regression	No support to the heterogeneous environment and unstable QoS	Scheduler is implemented
Energy-aware resource allocation algorithm [29]	Neural network	SLA nonviolation, no control wastage, and given no scalability	Cloud sim
Energy-efficient dynamic resource management [30]	Gradient boosting tree	Reduction in control utilization with the nonviolation of SLA	Cloud sim

**Table 2:** The abbreviation used in the proposed algorithm.

Name	Abbreviation
F_ev_	Feature value
S_l_	Significance level
Cm	Capsule model

**Table 3:** Accuracy (%) comparison.

Sr. no	Algorithm	Accuracy (%)
1	LR	70
2	PSO	76
3	Capsule network	85
4	CNN	94
5	Proposed CSLEC model	97

**Table 4:** Comparison of the number of trainable parameters and training time for the proposed model and other models.

Sr. no	Algorithm	Trainable parameters	Training time (ms)
1	LR	16896	588.31
2	PSO	17154	946.52
3	Capsule network	20960	967.14
4	CNN	33410	1702.43
5	Proposed CSLEC model	25346	1577.87

**Table 5:** The electric energy consumed by the considered servers at different levels of workload in watts (W).

Server capacity	0 (%)	10 (%)	20 (%)	30 (%)	40 (%)	50 (%)	60 (%)	70 (%)	80 (%)	90 (%)	100 (%)
Fujitsu M1	14.4	19.4	22.2	24.5	27.6	30.7	35.8	41.8	47.9	58.5	61
Fujitsu M3	13.5	17.8	20.5	22.5	24.5	27.2	30.8	35.9	42	48.2	52.3
Hitachi TS10	41	42.9	44.3	46.6	49.9	53.9	58.9	66.2	74.9	81.9	86.2
Hitachi SS10	37	39.9	42.3	44.8	47.4	50.5	54.2	59.9	65.3	68	70.8

**Table 6:** Computed results for Capsule algorithm.

Task	Arrival time	Processing time	Response time	Processor utilization	Energy consumption
T0	0	9	9	27	29.5
T1	1	3	2	13	14.1
T2	8	5	2	42	43.5
T3	16	2	15	53	54.7
T4	22	5	16	82	84.1

## Data Availability

The data used in this work are available at https://planetlab.cs.princeton.edu/datasets.html.
